The article "Extracellular matrix stiffness—The central cue for skin fibrosis" was published in 2023. Journal: Front Mol Biosci.

# Extracellular matrix stiffness—The central cue for skin fibrosis

**DOI:** 10.3389/fmolb.2023.1132353

**Published:** 2023-03-08

**Authors:** Kang Wang, Dongsheng Wen, Xuewen Xu, Rui Zhao, Feipeng Jiang, Shengqin Yuan, Yifan Zhang, Ya Gao, Qingfeng Li

**Affiliations:** ^1^ Department of Plastic and Reconstructive Surgery, Shanghai Ninth People’s Hospital, Shanghai Jiao Tong University School of Medicine, Shanghai, China; ^2^ Department of Burn and Plastic Surgery, West China Hospital, Sichuan University, Chengdu, Sichuan, China; ^3^ West China School of Medicine, Sichuan University, Chengdu, Sichuan, China; ^4^ School of Public Administration, Sichuan University, Chengdu, Sichuan, China

**Keywords:** skin fibrosis, extracellular matrix, stiffness, biomechanics, targeted therapy

## Abstract

Skin fibrosis is a physiopathological process featuring the excessive deposition of extracellular matrix (ECM), which is the main architecture that provides structural support and constitutes the microenvironment for various cellular behaviors. Recently, increasing interest has been drawn to the relationship between the mechanical properties of the ECM and the initiation and modulation of skin fibrosis, with the engagement of a complex network of signaling pathways, the activation of mechanosensitive proteins, and changes in immunoregulation and metabolism. Simultaneous with the progression of skin fibrosis, the stiffness of ECM increases, which in turn perturbs mechanical and humoral homeostasis to drive cell fate toward an outcome that maintains and enhances the fibrosis process, thus forming a pro-fibrotic “positive feedback loop”. In this review, we highlighted the central role of the ECM and its dynamic changes at both the molecular and cellular levels in skin fibrosis. We paid special attention to signaling pathways regulated by mechanical cues in ECM remodeling. We also systematically summarized antifibrotic interventions targeting the ECM, hopefully enlightening new strategies for fibrotic diseases.

## 1 Introduction

Dermal fibrosis is characterized by excessive deposition of ECM in the skin and belongs to a class of diseases caused by impaired tissue regeneration and faulty repair. It can occur in the normal repair of broken skin or as a significant hallmark in conditions such as systemic sclerosis (SSc) and keloids (Coentro et al., 2019). There are many diseases with this clinical manifestation of skin fibrosis. The etiology of these diseases varies and includes physical (radiation or mechanical stimulation), chemical, biological, and immune factors (Table 1; Figure 1). Numerous animal models have been developed and have been described in detail in Do NN’s review (Do and Eming, 2016).

The article "Extracellular matrix stiffness—The central cue for skin fibrosis" was published in 2023. Journal: Front Mol Biosci.

**TABLE 1:** Diseases with skin fibrosis symptoms.

Name of disease	Etiology	Clinical manifestation of skin	Biomarkers
Dermatofibroma (Wu, 2019)	Mild trauma such as an insect bite, related to genomic aberrations in 17q and 22q (Peng et al., 2022)	Hard solitary slow-growing papules (rounded bumps)	CD34 - (Bolognia et al., 2007)
		Appear in a variety of colors, usually brownish to tan	Stromelysin-3 + (Kim et al., 2007)
		Most often found on the legs and arms	Factor XIIIa + (Pierson, 2012)
			CD64 (Llamas-Velasco et al., 2022)
Scleroderma (Fett, 2013; Ota and Kuwana, 2021)	Autoimmune disease, caused by gene mutations (e.g., *DNASE1L3*, *STAT4*, HLA class II genes) or exposure to certain chemical compounds (e.g., silica, organic solvents)	Symmetrical skin thickening	Anti-scl70 (Kuwana et al., 2021)
		Skin stiffness increase	Anticentromere antibodies (Chung and Utz, 2004)
		Raynaud’s phenomenon	Anti-U3 (Peterson et al., 2016)
		Nail-fold capillary changes	Anti-RNA polymerase (Lazzaroni and Airò, 2018)
			Nucleolar antigens (Stochmal et al., 2020)
			CCL18 (Arron, 2021)
Keloids (Lee and Jang, 2018)	Related to skin tension, autoimmunity, genetic and epigenetic factors (such as HLA genes, TGF-β signaling pathway related genes) but not fully understood (Tsai and Ogawa, 2019)	Preferably in front of the sternum, earlobes, back, shoulders	STC2, SDC4, NOX4, DAAM1 (Yin et al., 2022)
		Firm, rubbery lesions or shiny, fibrous nodules	TNC (Xie et al., 2021)
		Sometimes producing a lump many times larger than that of the original scar	CD138 (Bagabir et al., 2016)
		Vary from red to dark brown in color	
		Sometimes accompanied by severe itchiness, pain, and changes in texture	
Hypertrophic scars (Lee and Jang, 2018)	Mechanical tension	Not extend beyond the boundary of the original wound	MiRNA-365a/b-3p (Lee et al., 2022)
	Inherited tendency (such as *ASAH1 g*ene, but not fully understood) (Santos-Cortez et al., 2017)	Not to the degree observed with keloids	Gal-1 (Kirkpatrick et al., 2021)
		May be itchy or painful	
		Often contain nerves and blood vessels	
		Develop after thermal or traumatic injury	
Dystrophic epidermolysis bullosa (Tartaglia et al., 2021)	Genetic defects within the human *COL7A1* gene	Highly susceptible to severe blistering	*COL7A1* (Pfendner et al., 1993)
		Chronic scarring	Tumor serine proteases C1r and C1s (Kopecki, 2020)
			HMGB1 (Petrof et al., 2013)
Porphyria cutanea tarda (Elder, 1998)	Inherited mutations	Individuals with PCT present with increasingly fragile skin on the back of the hands and the forearms. Other sun-exposed sites such as the face, scalp, neck, and arms may also be affected	Granular and homogeneous deposits of C5b-9 in vessels are characteristic immunofluorescence findings in patients with PCT (Vasil and Magro, 2007)
	Environmental impact		
Radiation dermatitis (Patel and McGurk, 2017; Yang et al., 2020)	Ionizing radiation, radiotherapy	Pain, sclerosis, hair loss and ulcers	StefinA3 and S100 calcium binding protein A8 (S100A8) (Huang and Glick, 2017)
	Some genes involved in the inflammatory pathway have been implicated in cutaneous radiation injury, such as *IL12RB2 rs3790568*	Advanced skin damage: dryness, scaly skin hyperpigmentation and loss of skin appendages	
Chronic Cutaneous Graft-Versus-Host Disease (Strong Rodrigues et al., 2018)	Graft rejection host: Bone marrow transplantation and other tissue transplantation	Flat moss-like lesions and polygonal papules in the early stages	ST2 (Srinagesh et al., 2019)
			REG3α(350)
		The skin becomes darker, atrophic and fibrotic, similar to scleroderma in late stages	TNFR1 (Pratta et al., 2022)
Nephrogenic Fibrosing Dermopathy (Woolen et al., 2020)	Renal failure	Patients present with hard, indurated, sometimes peau d’orange plaques	CD34, CD68 and factor XIIIa (Tsai et al., 2007)
Nephrogenic systemic fibrosis (Kaewlai and Abujudeh, 2012)	Unknown, possibly related to exposure to certain conventional gadolinium-containing contrast agents in magnetic resonance imaging	Swelling, tightness, red or dark patches, thickening and hardening of the skin of the trunk, burning, itching or severe tingling in the affected area	Fibroblast growth factor (FGF)23, osteoblast transcription factors Runt-related transcription factor 2, and osterix (Swaminathan et al., 2013)

The article "Extracellular matrix stiffness—The central cue for skin fibrosis" was published in 2023. Journal: Front Mol Biosci.

**FIGURE 1:** Relationship between the etiology, regulation mechanisms and targeted therapy of skin fibrosis. With environmental or genetic pathogenic factors, fibroblasts are activated and secrete large amounts of extracellular matrix. This process is further enhanced by the matrix stiffness upregulation. The TGF-β signaling pathway acts as the center of this positve feedback. Targeted therapies to break this vicious circle is a promising pathway in skin fibrosis treatment.

Not only in the skin, but fibrosis can also occur in almost all organs, such as the lungs, liver, kidneys and heart. There is broad agreement between the pathological mechanisms of different fibrotic diseases, but there are still differences. Skin fibrosis shares many signaling pathways with other organ fibrosis in the molecular mechanism, such as transforming growth factor-β (TGF-β) signaling pathway and Hippo signaling pathway. However, the skin is on the surface of the human body and is susceptible to mechanical stresses from internal or external actions of the body. Therefore, the mechanical stress-related regulation of skin is a direction of interest. Compared to other tissues in the body, it is easier for people to artificially modify the mechanical microenvironment of the skin to inhibit skin fibrosis, which could provide a new insight for the development of therapies related to skin fibrosis.

The article "Extracellular matrix stiffness—The central cue for skin fibrosis" was published in 2023. Journal: Front Mol Biosci.

Skin fibrosis is a public health issue for all humans, affecting more than 100 million people per year in developed countries, with a much higher prevalence in the worldwide population (Bayat et al., 2003). Skin fibrosis affects the normal physiological function of soft tissue and may also cause aesthetic problems and psychological distress (Bock et al., 2006). Despite the enormous market for anti-scar medications, estimated at over $12 billion annually in the United States (Sen et al., 2009), universally effective anti-scar treatment has been lacking thus far. How to reduce the occurrence of skin fibrosis, inhibit the progression of dermal and epidermal fibrotic diseases or even remove excess deposits of ECM in native tissues are significant concerns in the scientific and clinical fields. Elucidating the molecular mechanisms in the pathogenesis of skin fibrosis is crucial to developing therapeutic approaches.

The ECM is a collagen-based and well-organized dense meshwork of complex macromolecules containing proteins and polysaccharides secreted by resident cells such as fibroblasts. In addition to providing structural support for cells and tissues, the ECM has also been shown to significantly affect the proliferation, differentiation, and metabolism of parenchymal cells (Huang and Greenspan, 2012; Multhaupt et al., 2016; Tracy et al., 2016). There is clear evidence that ECM mechanical changes play vital roles in the occurrence and development of various kinds of skin fibrotic diseases, and increased ECM stiffness has been recognized as an important marker of fibrotic diseases (Hinz, 2009). Therefore, the mechanical properties of ECM have received increasing attention in the last decade. In the process of skin fibrosis, inflammatory cell infiltration, cytokine secretion, fibroblast proliferation and differentiation are the major biological events observed (Hsu et al., 2018). The combination of these events leads to ECM alterations in molecular composition and spatial structure, which is characterized as “ECM stiffness” from a macroscopic perspective. Altered ECM stiffness brings about changes in the extracellular mechanical microenvironment. The physical signals of matrix stiffening are sensed through receptors on the cell surface and further transduced intracellularly, triggering downstream signaling cascades and ultimately causing changes in transcription and posttranscription levels, leading to cellular metabolism and behavior alterations. Specifically, high ECM stiffness disrupts extracellular microenvironmental homeostasis, which is manifested by enhanced activation of mechanical signaling, increased levels of profibrotic cytokines, and consequently abnormally activated fibroblasts with promoted production of collagen fibers. Overall, this results in a positive feedback loop of “skin fibrosis–increased matrix stiffness–fibroblast activation–enhanced skin fibrosis” (Long et al., 2022). This loop accounts for the persistence and irreversibility of dermal fibrosis, making it a challenging and formidable task to inhibit the progression of skin fibrosis.

The article "Extracellular matrix stiffness—The central cue for skin fibrosis" was published in 2023. Journal: Front Mol Biosci.

This review systematically summarizes the interrelationship between ECM stiffness and skin fibrosis, in order of histologic, cellular and molecular levels (Figure 1). We focused on the cellular and molecular mechanisms of the pathogenesis of skin fibrotic diseases mediated by ECM stiffness, especially mechanotransduction and regulation.

## 2 ECM-related changes in skin fibrosis from the cellular and molecular perspectives

### 2.1 Histologic structure and mechanical microenvironment of skin tissue, and its changes during fibrosis

Mammalian skin mainly consists of three layers: the epidermis, the dermis, and the basement membrane (BM) that connects the epidermis and dermis (Fuchs and Raghavan, 2002; McGrath et al., 2004) (Figure 2A). The epidermis is composed of a keratinized stratified squamous epithelium that mainly contains keratinocytes in various developmental stages (McGrath et al., 2004; Rittié, 2016) (Figure 2A). Keratinocytes originate from the basal layer and become flattened dead corneocytes without a nucleus during maturation. During the maturation of keratinocytes, BM persistently produces new keratinocytes, pushing the old cells to the surface of the skin, which results in a stratum corneum with multiple layers of corneocytes on the surface of the skin. The main proteins expressed in different layers of the epidermis are also different (Bhattacharjee et al., 2019). Glycosaminoglycan (GAG) is the main component of epidermal ECM (Montagna et al., 1951), and includes hyaluronic acid (54%), heparan sulfate (33%) and chondroitin sulfate (13%) (Brown and Parkinson, 1983). In the stratum corneum, corneocytes act like bricks, while mixtures of extracellular lipids (ceramides, free fatty acids, and cholesterol) are similar to concrete, sticking the bricks together and conferring hydrophobic properties to the epidermis (Madison, 2003; McIntosh, 2003; Candi et al., 2005). The matrix components are highly organized, cross-linked, and closely integrated with keratinocytes. This matrix forms a barrier that resists mechanical stretching by external forces, reduces water loss from the body, and prevents invasion from pathogenic microorganisms (Cork, 1997; Holden et al., 2002; Baroni et al., 2012). Some studies found that initial stretching increased the proliferation of basal keratinocytes, leading to elongation of the basal layer and increased cellular density. The increased number of rete ridges suggests that they absorbed the impact of excessive proliferation, preserving the layered organization of the epidermis (Topczewska et al., 2019). In SSc, activated epidermal keratinocytes result in an increase in epidermal thickness (Nikitorowicz-Buniak et al., 2014; Russo et al., 2021). In atopic dermatitis, chronic skin injury causes hyperkeratosis of the epidermis in addition to dermal fibrosis (Lee et al., 2009). During the process of fibrosis, mechanical stimulation applied to the epidermis can be translocated to the dermis, activating fibroblasts by releasing cytokines such as connective tissue growth factor (CTGF or CNN2) and S100A9. This interaction demonstrates the integrity of skin structure and function (Nikitorowicz-Buniak et al., 2014).

The article "Extracellular matrix stiffness—The central cue for skin fibrosis" was published in 2023. Journal: Front Mol Biosci.

**FIGURE 2:** Schematic of skin histology viewed in cross-section. Three layers of mammalian skin: epidermis, basement membrane and dermis. **(A)** The epidermis contains corneocytes on the surface and keratinocytes in various developmental stages. The ECM molecules include GAG, hyaluronic acid, heparan sulfate, chondroitin sulfate and various kinds of extracellular lipids. The dermis consists of blood vessels and nerves. Many kinds of cells, including fibroblasts and macrophages, participate in the process of fibrosis. **(B)** and **(C)** The basement membrane is composed of individual laminin and collagen type IV, which provide mechanical connections between the epidermis and dermis.

The epidermal BM is a reticular complex composed of individual laminin or collagen type IV (Uitto et al., 1989), which provides mechanical connections between the epidermis and dermis through two structurally independent networks consisting of laminin 332, collagen type IV and XVII and laminins with α5-chains (Behrens et al., 2012) (Figures 2B,C). The epidermal BM plays a crucial role in skin fibrosis. The information transduction of the epidermis and dermis in both directions relies on specific structures on the BM, such as adhesive patches and hemi-bridging granules. In pathological cases, the damaged epidermis can also release inflammatory factors and chemokines, which cause a local inflammatory response in the skin and dermal inflammatory cell infiltration in the area covered by the epidermis. Nikitorowicz-Buniak et al. (2014) found that the number and size of basal cells in BM significantly increased in SSc compared to healthy tissue.

The article "Extracellular matrix stiffness—The central cue for skin fibrosis" was published in 2023. Journal: Front Mol Biosci.

The dermis is the inner layer of the skin, beneath the epidermis and BM. Compared with the epidermis, the dermis consists of blood vessels and nerves. The ECM is differentiated at different dermal levels and can be distinguished at the tissue level using histochemical staining, such as Herovici’s picropolychrome. Collagen, the most abundant protein in the dermal ECM, is secreted by fibroblasts and exists extracellularly as fibrin. The papillary dermis (PD) closest to the BM has a thin and loose arrangement of collagen fibers, which appear blue under Herovici’s picropolychrome staining; in the reticular dermis (RD), which is below the PD, collagen fibers are thicker and more densely arranged and stain purple (Watt and Fujiwara, 2011). The dermis is the main site of skin fibrosis. Using a combination of optical coherence tomography (OCT) and high-frequency ultrasound (HFUS) techniques, an increase in skin thickness during skin fibrosis was demonstrated (Ud-Din et al., 2019). Herovici staining demonstrated excessive collagen type III deposition in scar tissue and greater mechanical rigidity than normal tissue (Ud-Din et al., 2019). Elastin also undergoes significant changes during skin fibrosis, becoming broken in damaged skin, and is difficult to repair. Conversely, local tissue secretes more collagen, eventually leading to ECM stiffness (Wagenseil and Mecham, 2012). Furthermore, the molecular changes of the ECM during the fibrosis will be discussed later in Section 2.3. Interestingly, fibulin-5, an integrin-binding matricellular protein, can reduce tissue mechanical stiffness by promoting fiber assembly, as shown by the treatment of mice in a skin fibrosis model (Ikeda et al., 2009; Yanagisawa et al., 2009; Nakasaki et al., 2015). In normal tissue, the direction of collagen fiber is random (ultimately arranged in a mesh-like lattice under multiphoton microscopy) (Ueda et al., 2019).

The relationship between mechanical force and fibrosis was observed a long time ago. Although the detailed mechanism is unclear, antifibrotic therapy by modulating mechanical forces has been widely used in the clinic. In 1861, the anatomist Karl Langer summarized Dupuytren and Malgaigne’s earlier observations and pointed out that when puncturing cadaver skin with a conical spike, the puncture port was oval rather than circular (Carmichael, 2014). Further intensive puncturing of the skin surface and connecting the lines results in the formation of lines on the skin surface, now known as Langer’s lines (Abyaneh et al., 2014). This discovery helps reduce scar formation by making surgical incisions parallel to Langer’s lines (Paul, 2017). Langer’s lines also indicate the direction of maximum local skin tension, which is mainly affected by the arrangement direction of the main protein components of ECM, muscle contraction, and other factors (Silver et al., 2003; Bush et al., 2007; Casale et al., 2021). Ogawa et al. (2012) measured the distribution and skin stretching of 483 keloid patients and showed that mechanical force is an important factor driving keloid formation, even in genetically susceptible individuals. Hypertrophic scarring can be produced in experimental animal models by repeated mechanical force or sustained stretching at the incision edges (Shan et al., 2017). In addition, dilators are widely used in plastic and reconstructive surgery to obtain additional skin for grafting. This is because the continuous stretching force promotes the proliferation of the skin, including the ECM (Wang et al., 2015). In a large animal and phase I clinical study, Gurtner et al. (2011) showed that using a dynamic stress-shielding polymer device significantly reduced scar formation.

The article "Extracellular matrix stiffness—The central cue for skin fibrosis" was published in 2023. Journal: Front Mol Biosci.

### 2.2 Major cell types in skin tissue and their role in fibrosis

During skin fibrosis, abnormal changes occur in the number, variety, and metabolism of cellular populations, including resident cellular components and migratory cells in the skin (Smith and Chan, 2010; Deng et al., 2021). This process is often accompanied by changes in the cellular microenvironment, including mechanical properties and signaling molecular components of humoral components, and is observed macroscopically as immune inflammatory responses and immune cell infiltration (Pfisterer et al., 2021).

#### 2.2.1 Fibroblasts and myofibroblasts

Fibroblasts and myofibroblasts are key parenchymal cell populations, and they play significant roles in maintaining the homeostasis of the skin’s mechanical microenvironment under physiological conditions. When subjected to abnormal mechanical stimulation, however, excessive activation, hyperproliferation, and differentiation of fibroblasts can lead to excessive ECM deposition, which contributes to the progression of fibrosis and further leads to the formation of keloids, scars and SSc (Macarak et al., 2021) (Figure 3). Myofibroblasts are typically activated fibroblasts that can be transformed by soluble growth factors such as TGF-β and mechanical signaling (Elson et al., 2019). They are the most critical cellular populations in tissue remodeling and wound healing. Their main feature is the expression of smooth muscle actin, which enables contractility. Considering the tight junctions of myofibroblasts with ECM components, such as collagen, myofibroblasts can alter the mechanical properties of the local ECM and promote wound contraction and scar contracture. There is an intermediate stage called the proto-myoblast stage during the activation of fibroblasts (Watsky et al., 2010). The rate of transformation to proto-myoblasts is related to mechanical changes, such as the stiffness of the tissue. The stiffness is mainly influenced by external stretching forces and the contractile forces exerted on the ECM by the myofibroblasts, which leads to a positive feedback mechanism maintaining steady states of proto-myoblasts and myoblasts (Figure 3). The mechanical changes can also activate the secretion of TGF-β, a crucial factor during fibrosis; the detailed mechanism will be discussed in Section 3.2.1 and Figure 5. Fibroblasts and myofibroblasts can participate in ECM remodeling by secreting matrix metalloproteinases (MMPs) and tissue inhibitors of metalloproteinases (TIMPs). MMPs are endopeptidases, which are capable of ECM degradation and bioactive molecules processing. MMPs and TIMPs are important factors in skin ECM remodeling, which will be discussed in detail in Section 2.3.1 (Leong et al., 2021). Recent studies have shown that M2 macrophages promote fibroblasts to differentiate into myofibroblasts through an acid-sensing ion channel 3—macrophage colony-stimulating factor–TGF-β1 positive feedback loop in keloid patients. This further proves that the pathogenesis of skin fibrosis is not a single factor but the result of the long-term joint action of mechanical homeostasis and the inflammatory response in tissues (Wu et al., 2022) (Figure 4).

The article "Extracellular matrix stiffness—The central cue for skin fibrosis" was published in 2023. Journal: Front Mol Biosci.

**FIGURE 3:** The regulation in fibroblast activation. The fibroblasts derived from bone marrow can differentiate into an intermediate stage called protomyoblasts and then into myofibroblasts. Myoblasts can synthesize many kinds of molecules that contribute to mechanical changes in the ECM. In physiology, fibroblasts are vital to tissue homeostasis, while their excessive activation can lead to fibrosis in pathology. The rate of transformation to protomyoblasts and myofibroblasts is related to the mechanical changes in turn, which could lead to positive feedback. Mechanical changes can also activate the secretion of TGF-β, which is a crucial factor during fibrosis.

**FIGURE 4:** The positive feedback loop in skin fibrosis. ECM stiffness changes and inflammatory responses work together and lead to skin fibrosis. The mechanical property upregulation leads to the activation of TGF-β and other inflammatory factors. Inflammatory responses and inflammatory cell infiltration can promote the sedimentation of collagen and other ECM proteins. In general, a positive feedback loop in skin fibrosis is formed, and ECM stiffness plays a central role in this process.

The article "Extracellular matrix stiffness—The central cue for skin fibrosis" was published in 2023. Journal: Front Mol Biosci.

In addition to fibroblasts, myofibroblasts can also be derived from other cell types. Single-cell sequencing identified a bone marrow-derived fibroblast subgroup (Deng et al., 2021). Bone marrow-derived progenitor cells enter the bloodstream and circulate to specific tissues, where they colonize and further differentiate into fibroblasts that promote local collagen deposition, especially during wound repair (Fathke et al., 2004; Ishii et al., 2005; Suga et al., 2014; Sinha et al., 2018). Many recent studies have indicated that myofibroblasts in skin fibrosis can also be adipocyte-derived (El Agha et al., 2017) (Figure 3).

Fibroblasts exhibit functional diversity due to different origins, anatomical locations, and tissue microenvironments (Griffin et al., 2020). In skin tissue, fibroblasts perform functional diversity in different anatomical localizations and microenvironments (Driskell and Watt, 2015). Fibroblasts in the papillary layer play an irreplaceable role in forming hair follicles and PD, while fibroblasts in the reticular layer play an important role in developing the reticular layer and part of the subcutaneous tissue in the skin. After skin damage, reticulofibroblasts first migrate to the damaged site, producing a collagen-rich dermis, but the hair follicles cannot regenerate. In contrast, papillary fibroblasts are involved in wound healing at a later stage. The study of fibroblast heterogeneity can provide a better understanding of the differences between skin scarring and fibrosis after wound healing.

#### 2.2.2 Keratinocytes

Although ECM matrix thickening in skin fibrosis occurs mainly in the dermis, keratinocytes also play an important role in skin fibrosis. During wound healing and regeneration, keratinocytes migrate and proliferate at the wound edges at an early stage. Keratinocytes are observed to regulate fibroblast activation and ECM deposition by producing soluble inflammatory and growth factors in wound healing, hypertrophic scar formation, and other fibrotic processes (Shephard et al., 2004; Werner et al., 2007; Lee et al., 2019). In SSc, keratinocytes are found to promote fibroblast activation independent of TGF-β (McCoy et al., 2017). Keratinocytes can also modify the mechanical properties through the accumulation of collagen type I, increasing the expression of MMPs and decreasing the expression of tissue inhibitors of TIMPs (Russo et al., 2020).

Interestingly, keratinocyte proliferation, metabolism, and other cell behaviors are regulated by fibroblasts, forming a feedback loop. Fibroblasts inhibit keratinocyte apoptosis and promote keratinocyte survival and differentiation (El Ghalbzouri and Ponec, 2004; Peura et al., 2010; Fernandez et al., 2014). Fibroblasts also promote keratinocyte adhesion, possibly due to the secretion of soluble signaling molecules or transcription factors that freely diffuse to keratinocytes (Chowdhury et al., 2012; Quan et al., 2015; Yang et al., 2018).

The article "Extracellular matrix stiffness—The central cue for skin fibrosis" was published in 2023. Journal: Front Mol Biosci.

#### 2.2.3 Epithelial-mesenchymal transition (EMT)

EMT is the process by which epithelial cells lose polarity and acquire a mesenchymal phenotype. EMT can enhance cell migration, invasion capabilities, ECM matrix secretion, and antiapoptotic capabilities, making it an essential driver of tissue fibrosis (Kalluri and Neilson, 2003; Kalluri and Weinberg, 2009). EMT contributes to myofibroblast accumulation and increases myofibroblast contraction, migration, and ECM secretion ability. Integrin plays a significant role in fibrogenesis as a transmembrane receptor in EMT mediation and participates in the bidirectional signal transmission process between the external environment and cells (Yeh et al., 2012). Furthermore, evidence for microRNA-induced skin fibrosis *via* EMT is increasing. Some recent studies have shown that miRNA-21 and miRNA-200 increase the expression of the TGF-β type II receptor and contribute to EMT by interacting with the TGF-β pathway (Babalola et al., 2013). TGF-β can activate mesenchymal genes and inhibit epithelial gene expression through Smad or non-Smad signaling pathways, thus promoting the transdifferentiation of epithelial cells into mesenchymal cells (Derynck et al., 2014; Lamouille et al., 2014). Our research shows that additional stretching during skin regeneration can promote keratinocyte activation and EMT, suggesting that biomechanical force (BioF) can be a potential therapeutic target for skin fibrosis (Zhou et al., 2015).

#### 2.2.4 Immune cells and inflammatory responses

Immune cells are important regulators of ECM reconstruction. Activated immune cells can produce multiple cytokines, including TGF-β and nuclear factor kappa-B (NF-κB), which directly promote the activation of fibroblasts (Mack, 2018). The immune cells involved in this process are highly diverse, including macrophages, neutrophils, T cells, B cells, and natural killer cells (Huang et al., 2020). Different immune cells promote skin fibrosis by diverse mechanisms, but the mammalian target of rapamycin (mTOR) signaling pathway plays a central role in inflammation-mediated skin fibrosis (Yoshizaki et al., 2010). In addition, changes in the local immune microenvironment brought about by inflammatory cell infiltration are often accompanied by increases in the levels of various cytokines, such as IL-6 (interleukin-6), IL-17, and IFNs (interferon) (Brown and O’Reilly, 2019), and are involved in the pathogenesis of fibrosis by activating JAK-STAT signaling pathway regulation (Huang et al., 2020).

The article "Extracellular matrix stiffness—The central cue for skin fibrosis" was published in 2023. Journal: Front Mol Biosci.

Among the immune cells involved in fibrosis, macrophages have received the most extensive attention. Monocytes and macrophages are involved in the early response to inflammation (Guilliams et al., 2018). Macrophages can secrete tumor necrosis factor-α (TNF-α), TGF-β, interleukins (IL-1, IL-6, IL-8, IL-12), and various chemokines (Arango Duque and Descoteaux, 2014). Furthermore, these inflammatory factors can affect fibroblasts and promote ECM production (Yang and Plotnikov, 2021). Both M1 and M2 macrophages are involved in the development of fibrosis. M1 macrophages activate myofibroblasts by producing proinflammatory factors and chemokines (Braga et al., 2015). M2 macrophages mainly play an anti-inflammatory role but can produce TGF-β and promote ECM production (Mosser and Edwards, 2008; Sica and Mantovani, 2012). M2 macrophages promote wound healing and tissue regeneration after injury under physiological conditions. However, under pathological conditions, the stimuli that trigger the inflammatory response persist, and a large number of profibrotic factors, such as TGF-β and Galactin-3 secreted by M2 macrophages, play an important role in driving tissue fibrosis (Cao et al., 2014).

In addition, immune cells have been observed to directly interact with the ECM and actively participate in remodeling of the ECM. For example, macrophages release a variety of MMPs, such as MMP-10, MMP-12 and MMP-21, to promote ECM degradation (Skoog et al., 2006; Pellicoro et al., 2012; Feng et al., 2019). Th1 cells can secrete MMP-2 and MMP-9, enhancing the MMP secretion capacity of macrophages (Oviedo-Orta et al., 2008). Osteopontin (OPN), which contains an RGD motif and can bind to integrins, widely exists in the ECM (Oldberg et al., 1986). Macrophages, T cells, and NK cells can all express OPN (Murry et al., 1994; O’Regan et al., 1999) and further lead to skin fibrosis (Wu et al., 2012; Newe et al., 2021). In SSc, the overexpression of versican, which can bind to collagen type I and maintain the structural stability of ECM by CD14^+^ cells, is important for the formation of ECM stiffness (Masuda et al., 2013).

Mechanical forces and the immune system are dependent on each other. For example, the immune response is stimulated by increased ECM stiffness. Activated immune cells induce biomolecular secretion and lead to ECM stiffness increase directly or indirectly (Figure 4). Furthermore, mechanical stress can prolong the inflammatory response through a T-cell-dependent pathway, thereby promoting scarring (Wong et al., 2011). Prolonged changes in the immune microenvironment combined with changes in cellular mechanical stress lead to dysregulation of extracellular microenvironment homeostasis, ultimately leading to skin fibrotic lesions marked by excessive collagen deposition and ECM stiffness in the dermal ECM (Pakshir and Hinz, 2018; Pfisterer et al., 2021). In conclusion, during skin fibrosis, the positive feedback loop between ECM stiffness upregulation and immune activation is required for fibrogenesis and maintains the indispensable stimuli for fibrosis (Figure 4).

The article "Extracellular matrix stiffness—The central cue for skin fibrosis" was published in 2023. Journal: Front Mol Biosci.

### 2.3 Important biomolecules in ECM and their changes in fibrosis

The dermal matrix is a “fishnet-like” structure composed of a complex series of proteins, mainly containing collagen types I and III (Smith et al., 1982). Dermal ECM-specific proteins, including collagen type IX, collagen type XII, fibril-associated collagens with interrupted triple helices (FACIT) and small leucine-rich proteoglycan (SLRP), remodel the mechanical properties of the ECM by regulating protein crosslinking, participate in communication between cells and the matrix, regulate cell behavior and even determine cell fates (Chermnykh et al., 2018; Dengjel et al., 2020; Potekaev et al., 2021).

#### 2.3.1 Collagen and related regulatory proteins

Collagen is the most important component of skin ECM and the primary determinant of mechanical properties (Zhang et al., 1995; Ricard-Blum, 2011; Karayi et al., 2020). Collagen types I and III are the most abundant in the skin, and their gene transcription is significantly upregulated in fibrotic skin (Heino et al., 2009). Collagen type IV is the main component of BM (Ricard-Blum, 2011). Collagen types VI and VII help BM connect to the matrix of the papillary layer of the dermis by closely binding to collagen type I in the dermal matrix (Has et al., 2015). Collagen types IX and XII are fibrillar-associated collagens mediating collagen–collagen and collagen–other biomolecule connections. Collagen type XVII is a transmembrane collagen that regulates cell growth and metabolism (Has et al., 2015). Collagens can form a reticular structure that composes the main architecture of the ECM, mediates the communication between the ECM and cells, and participates in mechanosensitive signal transmission (Mak and Mei, 2017; Pozzi et al., 2017). FACIT, SLRP, and matricellular proteins can serve as molecular bridges that are important for the organization and stability of extracellular matrices. These molecules can effectively enhance the fibroblast response to TGF-β and regulate ECM stiffness by regulating fibril formation and collagen fiber cross-linking (Grässel and Bauer, 2013; Has et al., 2015; Chacón-Solano et al., 2022). In the development of skin fibrosis, ECM components change correspondingly. The expression levels of lumican and collagen type V were increased, while collagen fibril assembly was damaged (Zhou et al., 2021).

The article "Extracellular matrix stiffness—The central cue for skin fibrosis" was published in 2023. Journal: Front Mol Biosci.

Lysyl oxidase (LOX), mainly produced by fibroblasts, can mediate the cross-linking of lysine and hydroxylysine of different collagen peptides to form a stable collagen network (Vallet and Ricard-Blum, 2019; Vorstandlechner et al., 2020). Collagen is cross-linked by the deamination of lysine residues with the catalysis of LOX. The increased cross-linked form of collagen has higher mechanical strength and stronger resistance to MMP degradation (Clarke et al., 2013). Collagen matrices with increased hydroxyallysine cross-link levels were less susceptible to MMP-1 degradation than the collagen matrices containing low hydroxyallysine levels (van der Slot-Verhoeven et al., 2005). Correspondingly, the use of LOXL2/LOXL3 inhibitor can reduce collagen oxidation and collagen crosslinking, which represents an innovative therapeutic approach for the treatment of fibrosis (Schilter et al., 2019). Huang et al. (2019) found that TGF-β can mediate ECM stiffness through LOXs using two *in vitro* models containing fibroblasts from SSc patients. LOXs can also directly induce the production of ECM at the transcriptional level by changing the metabolism of fibroblasts, thus directly participating in the process of fibrosis (Nguyen et al., 2021). The increase was mediated by LOX-induced c-Fos expression, the nuclear localization of c-Fos, and the overexpression of IL-6 in fibroblasts.

MMPs are calcium-dependent zinc-containing endopeptidases. Dermal fibroblasts and leukocytes are the main sources of MMPs, especially MMP-2, which is usually secreted in the form of inactive proMMP (Wang, 2018). Many MMPs, such as MMP-1,2,3,8,11,13, are able to hydrolyze ECM proteins and reduce the stiffness of the ECM. TIMPs are natural inhibitors of MMP. TIMP and MMP work together to form proMMP-2/TIMP-2/3/4 and MMP-9/TIMP-1 that maintain the balance of ECM synthesis and degradation under physiological conditions (Vafadari et al., 2016; Cheng et al., 2017). In SSc, it was observed that the decreases in MMP-1 and MMP-3 expression and the increase in TIMP-1 expression resulted in the inhibition of the structural protein hydrolysis of ECM (Leong et al., 2021). MMP-13 is produced by fibroblasts in adult gums and fetal skin wounds and promotes rapid collagen remodeling and scar-free healing (Ravanti et al., 2001; Toriseva et al., 2012).

The article "Extracellular matrix stiffness—The central cue for skin fibrosis" was published in 2023. Journal: Front Mol Biosci.

#### 2.3.2 Integrins

Integrins are a family of transmembrane proteins (cell surface receptors) that mediate the interconnection between cells and the ECM. They mechanically anchor cells on the ECM and use their transmembrane structure to participate in the bidirectional signal transmission process between the external environment and cells (Henderson and Sheppard, 2013). Depending on their subtype, integrins have different functions, including collagen, laminin, leukocyte, and bilirubin receptors (Koivisto et al., 2018).

In addition to binding to the major structural proteins of the ECM, integrins can also bind to non-structural proteins such as a disintegrin and metalloproteinase (ADAM), thus directly contributing to the structural remodeling of the ECM (Watt and Fujiwara, 2011; Giebeler and Zigrino, 2016). Integrin can regulate ECM stiffness indirectly by activating latent TGF-β (Figure 5). The activated TGF-β induces the myofibroblastic differentiation. In addition, integrin contributes to autocrine TGF-β signaling (Asano et al., 2006a; Asano et al., 2006b). The integrin signaling pathway will be discussed in Section 4.2.

**FIGURE 5:** Integrin, Hippo and TGF-β signaling pathways mediate mechanical stress signaling to the cell. **(A)** TGF-β is secreted out of cells in an inactive form. Activated TGF-β can upregulate ECM stiffness through fibroblast activation. **(B)** Mechanical signals are involved in TGF-β activation.The interaction of activated TGF-β and TGFBR mediated the transmembrane transduction of ECM mechanical signals, which is transduced via two pathways, Smad and non-Smad, thereby regulating myofibroblast differentiation and the stiffness of the ECM. Integrins can signal through pathways such as FAK, ILK and Hippo, and there is crosstalk with the TGF-β pathway.

#### 2.3.3 Growth factors

Many studies have shown that growth factors are widely involved in the initiation of fibroblasts and the maintenance of a steady myofibroblast population during various fibrotic diseases. TGF-β is a crucial regulatory signaling molecule in fibrosis. TGF-β1 expression significantly increases in keloids, SSc, and skin fibrosis caused by radiation factors (Verrecchia et al., 2006; Verrecchia and Mauviel, 2007). Abnormally increased secretion of TGF-β leads to excessive collagen deposition and ultimately scar formation. TGF-β was also found to downregulate the expression of MMP-1 and upregulate the expression of TIMP-3 to inhibit the degradation of ECM (Edwards et al., 1987; Ihn, 2002; Leivonen et al., 2013).

Platelet-derived growth factor (PDGF) and connective tissue growth factor (CTGF) have also been found to play important roles in the progression of fibrosis (Ihn, 2002). In gene-edited mice overexpressing PDGF-α, excessive proliferation of fibroblasts, ECM deposition, and a fibrotic phenotype were observed in multiple organs and tissues. PDGF can be a downstream regulator of TGF-β and work synergistically with it in the process of fibrosis by binding with PDGFR (Olson and Soriano, 2009). PDGFRs are receptor tyrosine kinases that dimerize after ligand binding, activating the intracellular tyrosine kinase domains. These activated domains autophosphorylate several tyrosine residues, creating docking sites for signaling proteins and adaptors that are responsible for the signal transduction process attracting fibroblasts and macrophages.

The article "Extracellular matrix stiffness—The central cue for skin fibrosis" was published in 2023. Journal: Front Mol Biosci.

CTGF is induced by TGF-β and regulates fibroblast growth and ECM synthesis. CTGF is considered an important mediator in the pathogenesis of fibrosis and can strengthen the TGF-β/Smad3 signaling pathways (Verrecchia and Mauviel, 2007).

## 3 ECM stiffness acts as the central cue in skin fibrosis signaling network and contributes to the positive feedback loop in pathological conditions

With the reconstruction of ECM in fibrogenesis, the cells embedded in the matrix are constantly exposed to abnormal mechanical stress (Jansen et al., 2018; Potekaev et al., 2021). The behavior of cells is tightly controlled by the mechanical environment, which eventually leads to the activation of fibroblasts, excessive ECM accumulation and ultimately fibrosis. The initiation of fibrosis will start a positive feedback loop (Figure 4), in which the constantly increasing tissue stiffness will lead to the persistence and self-reinforcement of the fibrosis process. This hypothesis explains the continuation of fibrotic diseases observed clinically and the difficulty in reversing the trend of fibrosis.

### 3.1 Increased ECM stiffness modulates cell fate and function

The positive feedback loop between fibroblasts, myofibroblasts and mechanical stress was described in detail earlier in Section 2.2 and Figure 3. In addition, mechanical signals can transmit into cell directly by membrane proteins such as integrin and piezo1. The matrix stiffness increase can also indirectly activate parenchymal cells in ECM by inducing TGF-β activation (Figure 5). During skin fibrosis, immune cells are activated and can further modulate fibroblasts or participate in the fibrotic process by directly engaging in ECM alterations. This process is also a positive feedback loop (Figure 4).

#### 3.1.1 Immune cells

In the process of skin fibrosis, changes in ECM structure and composition regulate the activation of immune cells and induce immune cell infiltration (Lu et al., 2011; Hallmann et al., 2015; Simon and Bromberg, 2017). The proteolytic products of ECM proteins, including collagen, elastin, laminin, and hyaluronic acid, can act as inflammatory mediators (Adair-Kirk and Senior, 2008). Neutrophils bind to the 7S domain of collagen type IV through surface receptors. It is suggested that neutrophils may have chemotaxis to the collagen type IV hydrolyzed region *in vivo* (Senior et al., 1989). In addition, the mechanical force can act directly on immune cells and participate in the activation and aggregation of immune cells in fibrosis (Figure 4).

The article "Extracellular matrix stiffness—The central cue for skin fibrosis" was published in 2023. Journal: Front Mol Biosci.

T and B cells perceive the mechanical microenvironment through mechanically sensitive T-cell receptor (TCR) and B-cell receptor (BCR) or antigen-presenting cell (APC) interactions (Huse, 2017; Saitakis et al., 2017). In 2D cell culture, the enhancement of culture surface rigidity can promote the activation, migration and proliferation of T cells (O'Connor et al., 2012). The sensing of mechanical signals may be related to CD3 (Judokusumo et al., 2012). CD3 (ε chain) can be attached to polymers under costimulation by CD28 (Riha and Rudd, 2010) and presented to primary T cells. Many proteins involved in this process, including interleukin-2 (IL-2) secretion and proliferation, interact directly or indirectly with the actin cytoskeleton for signaling (Bashour et al., 2014).

In addition, Majedi et al. found that in 3D cultured T cells, an ECM environment with a high elasticity modulus induced the expression of inflammatory factors such as IL-2, IFN-γ and TNF-α (Majedi et al., 2020). The enrichment of inflammatory factors can further induce tissue fibrosis. Yes-associated protein 1 (YAP), a well-established mechanosensitive protein, has also been found to play an important role in mechanical signal transduction between T cells and the ECM (Meng et al., 2020). Regulation of T-cell metabolism is mainly attributable to nuclear factor of activated T cells (NFAT)-driven transcription. YAP is expressed in activated T cells and negatively regulates T-cell proliferation and activation in response to the mechanical microenvironment by directly restricting NFAT1 translocation to the nucleus (Meng et al., 2020). However, YAP does not affect the early activation of T cells (Meng et al., 2020). We will discuss YAP-related signaling processes in detail in 4.2.3. Zeng et al. (2015) have shown that the rigidity of the substrate cultured in 2D can regulate the proliferation of B cells. The increase in matrix stiffness can promote or inhibit the proliferation of B cells, which is different in response to different proliferation stimuli. Macrophages have also been demonstrated to be regulated by mechanical signals. Under low substrate stiffness, the expression of CD86 on the cell surface of bone marrow-derived macrophages (BMMs) increased and secreted more proinflammatory factors, such as IL-1β and TNF-α. With increasing ECM stiffness, the expression levels of CD206, IL-4 and TGF-β in BMMs increased accordingly, while the synthesis of ROS decreased (Chen et al., 2020). In addition, the increase in matrix stiffness increases its migration capability (Hind et al., 2015), which is regulated by the PI3K-AKT1 and Rac signaling pathways. YAP-mediated mechanical transduction is also involved in macrophage-dependent inflammation (Meli et al., 2020).

The article "Extracellular matrix stiffness—The central cue for skin fibrosis" was published in 2023. Journal: Front Mol Biosci.

Similarly, the mechanical properties of the matrix can affect neutrophil adhesion, diffusion and migration (Oakes et al., 2009). The difference in ECM stiffness leads to the migration of neutrophils to sites of injury. The magnitude of ECM stiffness determines the neutrophil migration rate and the final diffusion area (Oakes et al., 2009). Neutrophils migrate more slowly on harder substrates, but neutrophils eventually move farther, considering the longer migration duration (Oakes et al., 2009).

The increased matrix stiffness also enhanced the proinflammatory function of dendritic cells (DCs), and the glycolysis of DCs was enhanced to meet the energy requirements of DC activation and the raw material requirements for biosynthesis (Chakraborty et al., 2021). Zeng et al. (2015) also found that DCs receive extracellular mechanical signals through multiple signaling pathways. The Hippo signaling pathway is involved, as it has been shown that the Hippo signaling molecule MST1/2 regulates DC metabolism (Du et al., 2018). At the same time, DCs may mediate the transcription of target genes in response to substrate stiffness by upregulating the expression of the transcriptional coactivator with PDZ-binding motif (TAZ) gene and its Hippo signaling partner YAP and its translocation into the nucleus (Chakraborty et al., 2021).

#### 3.1.2 Stem cells

Matrix stiffness can be used as an effective regulator for stem cells (Chermnykh et al., 2018). Studies by Engler et al. (2006) have shown that different levels of ECM stiffness can guide mesenchymal stem cells (MSCs) to differentiate into osteoblasts, myocytes, and nerve cells. This may be related to the anchoring density and anchoring force between stem cells and ECM (Park et al., 2011; Trappmann et al., 2012). The directional differentiation of tissue-resident MSCs is one of the important sources of myofibroblasts (Kramann et al., 2015). Continuous culture of MSC renewal on hydrogel with a rigid gradient of 1.0 ± 0.1 kPa/mm showed that MSCs migrated to a more rigid matrix (Tse and Engler, 2011). In addition, increased stiffness of the ECM induces EMT, indicating that epithelial cells can transdifferentiate into myofibroblasts by high mechanical stress (Leight et al., 2012).

The article "Extracellular matrix stiffness—The central cue for skin fibrosis" was published in 2023. Journal: Front Mol Biosci.

### 3.2 Increased ECM stiffness activates fibrosis-related signaling biomolecules

#### 3.2.1 TGF-β is directly and indirectly modulated by mechanical signals

We previously discussed the upregulation of ECM stiffness by TGF-β in detail (Section 2.2.1; Figure 3). Mechanical stress also has a regulatory effect on TGF-β, which forms a positive feedback loop. The mechanical properties of the ECM have an important impact on the activity and availability of TGF-β1. Mature TGF-β is a covalent homodimer. Its precursor protein is processed intracellularly after translation and cleaved to form latency-associated peptide (LAP) and mature TGF-β. LAP forms a complex with TGF-β in a non-covalently bound form and masks the active site of TGF-β. TGF-β is activated by dissociating LLC bound to LAP and/or ECM. This process can occur through various mechanisms, including integrin-LAP interaction-mediated TGF-β activation and mechanical tension-induced TGF-β activation (Mu et al., 2002; Frangogiannis, 2020) (Figure 5A). Pierre-JeanWipff et al. also found that myofibroblast contraction can directly activate TGF-β1 stored in the ECM (Wipff et al., 2007).

#### 3.2.2 Integrins mediate mechanical signal transduction and TGF-β activation

Integrin plays a central role in the activation of TGF-β during fibrosis (Henderson et al., 2013) (Figure 5B). Through the structural analysis of integrin and TFG-β, Ruoslahti and Pierschbacher et al. showed that TGF-β1 and TGFβ-3 bind to integrin based on their linear sequences of arginine, glycine, and aspartic acid (RGD sequence) (Ruoslahti and Pierschbacher, 1987) (Figure 5B). Munger’s research in the SSc mouse model showed that fibroblasts upregulated the expression of αvβ5 vitronectin receptor and led to the activation of latent TGF-β (Munger et al., 1999). Like many other ECM protein components, LAP contains RGD motifs that can be specifically bound by integrins. In addition, integrin αvβ8 activates by presenting the potential TGF-β complex to MMPs, resulting in the release of free TGF-β into the extracellular environment (Prieto et al., 1993). In mice, knockout of integrin subunits (β6, αv and β8) can activate TGF-β1 (Huang et al., 1996; Bader et al., 1998; Zhu et al., 2002), and mutations in the integrin binding sites in LAP produced the same effects as TGF-β1 knockout (Shull et al., 1992; Yang et al., 2007; Hinz, 2015).

## 4 ECM stiffness-mediated mechanical signaling pathway

Various signaling molecules, including integrins and TGF-β, can mediate mechanotransduction. Once the signal is transduced across the membrane into the cytoplasm and nucleus, it will cause a series of downstream changes (Figure 5). Figure 5B shows the complicated relationship among several most important signaling pathways.

The article "Extracellular matrix stiffness—The central cue for skin fibrosis" was published in 2023. Journal: Front Mol Biosci.

### 4.1 TGF-β signaling pathway

The secretion and activation of TGF-β are regulated by immune cells and the extracellular mechanical microenvironment. Activated TGF-β binds to transforming growth factor-β receptor (TGFBR) on the surface of fibroblasts, upregulating α-SMA expression and promoting collagen secretion and cell proliferation. In addition, TGF-β acts as an inflammatory factor, inducing an inflammatory response (Li and Flavell, 2008) and indirectly promoting local tissue fibrosis. In skin fibrosis, the most classical signaling pathway is achieved by activating Smad transcription factors by TGFBR (Figure 6). TGF-β can also activate other proteins, such as Ras and Rho protein-mediated signaling pathways, called non-Smad signaling pathways (Figure 5).

**FIGURE 6:** Interaction of the TGF-β signaling pathway through Smad and non-Smad pathways in fibrosis. Mature TGF-β binds to TGFBR and acts on downstream molecules through the Smad and non-Smad pathways, thereby regulating ECM production. The downstream molecules of these pathways can interact with the molecules of the Smad pathway to inhibit or promote ECM production.

TGFBR has serine/threonine kinase activity and is activated upon binding to TGF-β, mediating different downstream signaling pathways through the phosphorylation of different substrates within its cells and ultimately resulting in phenotypic alterations, including fibroblast activation and EMT (Lamouille et al., 2014). The abundance of TGFBR in cell membrane species, including NIH-3T3 fibroblasts, can be regulated by endocytosis (Vander Ark et al., 2018). TGFBR is thought to be brought into the cell by endocytosis along with the cell membrane to form endocytic vesicles. Liposomes containing TGFBR can also bind to the cell membrane again and rapidly increase the cellular sensitivity to TGF-β (Huang and Chen, 2012).

TGFBR, a specific receptor of the TGF-β family, is divided into three types: TGFBR1, 2, and 3. TGFBR1 and TGFBR2 form stable complex receptor tetramers in the presence of TGF-β. First, TGF-β binds to TGFBR2 and activates its phosphokinase activity. Subsequently, TGFBR2 phosphorylates TGFBR1 (Budi et al., 2017; Yan et al., 2018) (Figure 6). TGFBR1 then phosphorylates R-Smads, after which the signal is transmitted intracellularly through the Smad signaling pathway and ultimately regulates the transcription of specific genes. TGFBR3 has no kinase activity but can present TGF-β to TGFBR2 and stabilize the complex between TGFBR1 and TGFBR2 (López-Casillas et al., 1993; Bilandzic and Stenvers, 2011). TGFBR3 is particularly important for TGF-β2 signaling (Kim et al., 2019; Kudipudi et al., 2019). However, the formation of the complex between TGFBR1 and TGFBR2 is inhibited when TGFBR3 alone binds to TGFBR1 or TGFBR2, thereby suppressing TGF-β-mediated Smad signaling (Tazat et al., 2015). In addition, the extracellular structural domain of TGFBR3 can be detached from the cell membrane, and further binding to TGF-β can block signal transduction into the cell (López-Casillas et al., 1994) (Figure 5B).

The article "Extracellular matrix stiffness—The central cue for skin fibrosis" was published in 2023. Journal: Front Mol Biosci.

The Smad pathway regulates the production of the ECM matrix together with the non-Smad pathway. Collectively, there is crosstalk between the Smad and non-Smad pathways of TGF-β. For example, R-Smads are phosphorylated at multiple sites by other kinases (MAPKs, CDK2/4, and ROCK). The activity of R-Smads is finely regulated and accomplishes the integration of different signaling inputs (Wrighton et al., 2009; Liu and Feng, 2010). The proteins mentioned above involved in regulating R-Smads are regulated by the non-Smad pathway and act as substrates of the non-TGF-β signaling pathway. In addition, TGF-β-mediated downstream factors can act synergistically with signaling cascades such as Wnt and Notch (Derynck and Zhang, 2003). Thus, the decision to develop fibrotic disease results from a combination of different signals, not from a specific pathway alone, which is consistent with the fundamental laws of life.

In conjunction with the Smad and non-Smad pathways, TGF-β promotes the secretion of collagen type I, collagen type II, and fibronectin by fibroblasts in the human dermis (Varga et al., 1987). Posttranslational transport and modification of collagen are also extensively regulated by TGF-β, including proteins such as HSP47, PLOD2, and P4HA3 (Ishida and Nagata, 2011; Bourhis et al., 2012; Ishikawa and Bächinger, 2013). Extracellular meprin and LOX are involved in collagen maturation assembly. These two proteins are abundantly expressed at fibrotic sites and are induced by TGF-β (Broder et al., 2013; Biasin et al., 2014; Laczko and Csiszar, 2020). TGF-β also induces the expression of protease inhibitors, such as TIMP, and inhibits ECM hydrolysis (Edwards et al., 1987).

#### 4.1.1 Smad signaling pathway

Smads are a family of structurally similar proteins that are the main carriers of intracellular signaling of the TGFBR (Itoh et al., 2000; Attisano and Tuen Lee-Hoeflich, 2001) (Figure 6). Smads can be classified into three subtypes based on their function, namely, receptor-regulated Smads (R-Smads), cochaperone Smads (Co-Smads), and inhibitory Smads (I-Smads) (Figure 5). Smads 1, 2, 3, and 5 and Smad8 are R-Smads located mainly in the cytoplasm and can be activated by phosphorylation of TGFBR. R-Smads can bind to specific DNA sequences or G/C-rich DNA regions (Shi and Massagué, 2003). Cooperating transcription factors can help stabilize Smad binding to DNA and enhance their specificity in recognizing DNA sequences. Smad4 is the only known Co-Smad expressed in humans and binds to activated R-Smads to cross the nuclear membrane. The remaining two Smads, Smad6 and Smad7, are mainly located in the nucleus and move to the plasma membrane in response to TGF-β stimulation. Activated Smad7 can bind to activated TGFBR to inhibit the phosphorylation of R-Smads (Shi and Massagué, 2003). I-Smads can also block TGF-β downstream signaling by preventing the nuclear translocation of R-Smads (Verrecchia et al., 2006; Verrecchia and Mauviel, 2007). In addition, Smad7 can act as an articulatory protein that promotes the binding of TGFBR1 to E3 ligases, thereby mediating the degradation of TGFBR1 *via* the ubiquitin pathway (Vander Ark et al., 2018).

The article "Extracellular matrix stiffness—The central cue for skin fibrosis" was published in 2023. Journal: Front Mol Biosci.

Smad3 appears to be a key component of the signal transduction pathway involved in the fibrosis process. Smad3-deficient mice were found to be protected from radiation-induced skin fibrosis (Flanders, 2004). Using a combinatorial cDNA microarray promoter transactivation approach, Franck Verrecchia et al. identified Smad3/4 gene targets in cultured dermal fibroblasts: COL1A1, COL3A1, COL5A2, COL6A1, COL6A3, and TIMP-1 (Verrecchia et al., 2001). Thus, the TGF-β/Smad signaling pathway is essential for activating skin fibrillar collagen genes.

The Smad signaling pathway promotes the expression of proteins such as JunB (Jonk et al., 1998), PDGF (Taylor and Khachigian, 2000), and integrin, thus indirectly regulating the process of tissue fibrosis (Figure 5). In addition, the TGF-β/Smad signaling pathway inhibits the degradation of the ECM. The TGF-β/Smad signaling pathway also inhibits the transcription of MMP-1 (Yuan and Varga, 2001) and activates the expression of human plasminogen activator inhibitor-type 1 (PAI-1) (Dennler et al., 1998).

#### 4.1.2 Non-smad signaling pathways

##### 4.1.2.1 Ras/Raf/MEK/ERK pathway

Ras is a small G protein that can hydrolyze GTP to GDP and then rebind to GTP with the assistance of guanine nucleotide exchange factor (GEF) and GTPase-activating protein (GAP). The different binding substrates result in two distinct states of Ras, which act as a switch in intracellular signal transmission. When Ras binds to GTP, the signaling pathway is “on”. When RAS hydrolyzes GTP to GDP, the signaling pathway is “off”. TGF-β1 increases mRNA levels and exogenous Ras promoter activity, thereby stimulating Ras (Brabletz and Brabletz, 2010; Su et al., 2020). Activated Ras activates Raf, which further activates mitogen-activated protein kinase kinase (MEK or MAPKK) and triggers a cascade reaction. Together, the proteins involved in this process form the Ras/Raf/MEK/extracellular signal-regulated kinase (ERK) signaling pathway (Figures 5, 6).

The article "Extracellular matrix stiffness—The central cue for skin fibrosis" was published in 2023. Journal: Front Mol Biosci.

An essential feature of tissue fibrosis is the occurrence of EMT (Lamouille et al., 2014). Activation of the ERK signaling pathway is required for TGF-β-induced EMT (Xie et al., 2004). TGF-β can activate the ERK pathway through upstream factors (e.g., Ras/Raf) and through more downstream factors (e.g., MEK) (Xie et al., 2004). The ERK signaling pathway can lead to overexpression of FOXM1 at the protein and mRNA levels, which in turn leads to indirect upregulation of EMT-related transcription factors (e.g., ZEB1 and ZEB2) and induction of the EMT process by the downregulation of microRNA-200b (Brabletz and Brabletz, 2010).

Ras affects TGF-β Smad signaling mainly by regulating the activation level of Smad2/3 (Figure 6). Ras interacts with SPSB1, a negative regulator of TGFBR2 on the cell membrane, to promote the degradation of the SPSB1 protein. Decreased levels of SPSB1 stabilize TGFBR2, thereby enhancing Smad2/3 phosphorylation and signaling (Burch et al., 2010; Liu et al., 2018). Activation of ERK can increase or decrease Smad signaling (Adhikari et al., 2007; Lei et al., 2019). Ras can inhibit BMP-induced nuclear accumulation of Smad1 at four sites in the junctional structural domain (Kretzschmar et al., 1999). Through PI3K, Pak2 activation can lead to cell type-dependent activation of ERK (Hough et al., 2012) (Figure 5). This activated ERK phosphorylates Smad2 primarily within its junctional region, leading to Smad-mediated transcriptional activation. This phosphorylation process occurs mainly in the nucleus by Smad2.

##### 4.1.2.2 TAK1-related pathway

TGF-β-activated kinase 1 (TAK1) is a member of the mitogen-activated protein kinase kinase kinase (MAPKKK) family (Xu and Lei, 2020). Activating TAK1 by TGF-β acts upstream of NF-κB and mitogen-activated protein kinases (MAPKs), thereby regulating ECM. Dynamic regulation of ubiquitination and deubiquitination plays an important role in TAK1-mediated activation of NF-κB (Lei et al., 2019). TRAF6 and TRAF4 are ubiquitin ligases (E3) (Figure 5). Upon induction of TGFBR, TRAF6/TRAF4 undergoes autoubiquitination and activates nuclear factor NF-κB *via* the cytokine interleukin 1 (Xie et al., 2004; Brabletz and Brabletz, 2010). After the recruitment of the bridging protein TAB1, TAK1 is autophosphorylated. It can affect the NF-κB pathway by regulating the IkappaB kinase (IKK)-subunit NFκB essential modulator and the NFκB-activating kinase IKKβ (Adhikari et al., 2007; Lei et al., 2019) (Figure 6).

The article "Extracellular matrix stiffness—The central cue for skin fibrosis" was published in 2023. Journal: Front Mol Biosci.

The MAPK pathway is activated by the phosphorylation of TAK1 through a cascade reaction (Fang and Richardson, 2005) (Figure 6). MAPKs are a large family of serine-threonine kinases with three main subfamilies: ERKs, c-Jun N-terminal kinases (JNKs) or stress-activated protein kinases (SAPKs) and p38 MAPKs. JNK can also be regulated by the activation of TAK1 (Sorrentino et al., 2008) (Figure 6). Activation of both JNK and p38 is not Smad dependent (Yamashita et al., 2008). In fibroblasts, activation of JNK inhibits TNF-induced apoptosis (Ventura et al., 2004). Knockdown of focal adhesion kinase (FAK) in fibroblasts in mice and modeling of hypertrophic scar models revealed significant reductions in inflammatory responses and fibrosis in mice. In addition, JNK can induce fibrosis by stimulating the inflammatory response. This process involves the activation of AP-1 and NF-κB and the transcriptional upregulation of inflammation-related genes (Ip and Davis, 1998; Workman and Habelhah, 2013). Activation of p38 MAPK plays an important role in the differentiation of fibroblasts into myofibroblasts, and this process is regulated by mechanical signaling. p38 MAPK promotes the expression of collagen type I (Sato et al., 2002), and p38 inhibitors abrogated the upregulated expression of collagen type I in fibroblasts with SSc disease (Ihn et al., 2005; Matsushita et al., 2017).

Activation of p38 MAPK plays an important role in the differentiation of fibroblasts into myofibroblasts, and this process is regulated by mechanical signaling. Studies have shown that inhibition of p38 can downregulate the expression of myofibroblast-related genes (e.g., ED-A fibronectin) and genes encoding LOX, thereby inhibiting collagen maturation and reducing ECM. In contrast, culturing fibroblasts with p38 inhibitors inhibits their activation process (Dolivo et al., 2019). In addition, p38 transduces mechanical signaling *via* the transcription factor serum response factor (SRF) and phosphatase to differentiate fibroblasts (Wang et al., 2022). These effects can be replicated in several primary human dermal fibroblast cell lines. Stem cells of adipose tissue origin can inhibit hypertrophic scarring by downregulating p38 expression (Li et al., 2016a). Overall, JNKs and p38 MAPKs can exert antagonistic effects on cell proliferation and survival, depending on the type of cell, the strength of the signal, the duration of the signal, and the crosstalk between different signals (Wagner and Nebreda, 2009). JNK and p38 MAPK pathways regulate the activity and expression of key inflammatory mediators, which allows them to be potent promoters of fibrosis (Wagner and Nebreda, 2009).

The article "Extracellular matrix stiffness—The central cue for skin fibrosis" was published in 2023. Journal: Front Mol Biosci.

A link between the p38/JNK and Smad pathways was established through the interaction between TAK1 and I-Smads (Figure 6). Smad6 inhibits TGF-β-induced activation of the TAK1-related signaling pathway, which occurs by blocking the ubiquitination of TRAF6 (Jung et al., 2013). Smad7 promotes TGF-β downstream of JNK and p38 MAPK activation (Mazars et al., 2001; Edlund et al., 2003). Specifically, Smad7 may direct TGF-β receptors to lipid rafts where TRAF6 is located, promoting TAK1 and downstream p38/JNK activation (Zhang, 2017). JNK and p38 signaling pathways have a facilitative effect on the Smad signaling pathway. In activated hepatic stellate cells, JNK in the TGF-β pathway can induce Smad2/3 phosphorylation (Yoshida et al., 2005). Similarly, p38 in rat myofibroblasts can phosphorylate Smad3 (Furukawa et al., 2003).

##### 4.1.2.3 PI3K-AKT pathway

TGF-β has also been shown to activate AKT *via* PI3K and lead to EMT and cell migration. This process is not dependent on Smads (Bakin et al., 2000) (Figures 5, 6). In addition to TGFBR, AKT can also be activated by ubiquitinated TRAF6 (Yang et al., 2009). This suggests that TRAF6 can indirectly activate AKT through TGFBR activation.

The mTOR can be activated specifically by AKT. It can promote EMT and increase cell size and protein content, migration, and invasion (Lamouille and Derynck, 2007). In cancer cells, the TGF-β/PI3K/AKT pathway can activate mTOR complex 1 (mTORC1), mTOR complex 2 (mTORC2), and S6 kinase, thus promoting EMT (Lamouille et al., 2012). Considering that mTORC2 contributes to enhancing Akt activation, there is positive feedback in PI3K-AKT pathway (Lamouille et al., 2012) (Figure 6). The TGF-β/PI3K/AKT signaling pathway induces fibroblast proliferation and conversion to myofibroblasts (Wilkes et al., 2005). A complex regulatory relationship exists between AKT and Smads (Zhang, 2017).

##### 4.1.2.4 GTPases downstream of TGF-β

TGF-β can activate Rho-like GTPases in a cell type-dependent manner, leading to key events in EMT, such as cell adhesion and cell migration (Mu et al., 2012). The Rho GTPase family, which includes RhoA, RhoB, Rac and Cdc42, is involved in many actin-related cellular processes to complete nuclear signaling (Phuyal and Farhan, 2019). TGF-β triggers the degradation of Rho through ligand-triggered TGFBR2 action, causing degradation of Rho, leading to direct phosphorylation of Par6 and promoting the recruitment of the ubiquitin ligase Smurf1, which targets RhoA for degradation (Zhang et al., 2004; Sutariya et al., 2016). The tumor microenvironment plays a crucial role in promoting EMT by controlling the subcellular localization and downstream signaling of Rac1/Cdc42 and Rac1b (Kalli et al., 2022). At the same time, TGF-β can activate RhoA independently of Smad2/3, leading to the activation of Rho-associated coiled-coil-containing protein kinase (ROCK) and EMT (Bhowmick et al., 2001) (Figure 6). ROCK phosphorylates myosin phosphatase, thereby inhibiting its phosphatase activity, leading to increased levels of phosphorylated myosin and induction of actomyosin-based contraction (Harvey et al., 2004).

The article "Extracellular matrix stiffness—The central cue for skin fibrosis" was published in 2023. Journal: Front Mol Biosci.

In addition, there may have an interaction between Cdc42 and the TGF-β receptor complex (Barrios-Rodiles et al., 2005) (Figure 6). TGFBR3 is often considered to be a coreceptor that activates Cdc42 through interaction with the scaffolding protein β-arrestin2 and is presented to its signaling receptor (Mythreye and Blobe, 2009). Cdc42 can bind to p21-activated kinase 2 (PAK2) and induce PAK2 conformational changes, which lead to PAK2 activation. Furthermore, PAK2 blocks Smad2 and Smad3 activation in a kinase activity-dependent manner (Figure 6). Phosphorylation of Ser-417 on Smad2 by PAK2 inhibits the interaction of Smad2 with TGFBR1 (Yan et al., 2012).

### 4.2 Integrin signaling pathway

Integrin β1 (ITGB1), also known as CD29, binds to integrins α1 and α2 to form integrin complexes, which are transmembrane collagen receptors. Within the cytoplasm, integrins bind to the actin cytoskeleton. Thus, integrins firmly attach the cytoskeleton to the ECM and promote cell adhesion.

Integrins can bind to many substrates in ECM. ITGB1 forms a heterodimer with integrin α3, which acts as a receptor for netrin-1 and reelin in the ECM. Kim and others showed that integrin α3β1 forms a complex at the apical junction with the TGFBR1 receptor and E-calmodulin. Upon TGF-β stimulation, integrin α3β1 triggers the formation of the pY654-β-catenin/pSmad2 complex and then upregulates EMT-related downstream gene expression (Kim et al., 2006; Kim et al., 2009a; Kim et al., 2009b). Numerous studies have shown that integrins αvβ3, αvβ5, αvβ6, and αvβ8 can bind to RGD sequences in LAP, thereby promoting the activation of latent TGF-β (Munger et al., 1999; Mu et al., 2002; Asano et al., 2006c; Henderson and Sheppard, 2013) (Figure 5B).

Integrins can directly participate in the downstream transduction of mechanical signals, ultimately regulating matrix remodeling, cell migration, and angiogenesis (Harburger and Calderwood, 2009). It is generally accepted that integrin α subunits are involved in extracellular to intracellular signaling, whereas β subunits are involved in intracellular to extracellular signaling (Hynes, 2002). Specifically, the process of β-subunit regulation is one in which intracellular signals modulate integrins to cause conformational changes in their extracellular structure, thereby increasing their affinity for extracellular ligands (Zhao et al., 2016). The cellular state receives regulation that can alter the affinity to the ECM and thus regulate the mechanical state (Figure 5B).

The article "Extracellular matrix stiffness—The central cue for skin fibrosis" was published in 2023. Journal: Front Mol Biosci.

Talin, a cytoskeletal protein, is essential in integrin activation (Calderwood, 2004). Talin is concentrated in areas of cell-matrix intercontact, such as adhesive patches, and connects integrins to the actin cytoskeleton (Figure 5B). Each subunit consists of an amino-terminal head and a carboxy-terminal rod-like tail. The heads of these subunits can bind to integrins, while the tail contains an actin-binding site that binds directly to actin. Talin can be joined head to tail, creating a state of self-activated inhibition. Interestingly, integrin α and β subunits are close to each other in the quiescent state, forming a low ligand affinity conformation. Talin conformational changes are induced by PIP2 *via* charge action, leading to the direct binding of talin to the integrin β subunit (Wang, 2012). In the case of indirect binding, talin binds and activates PIPKIγ, which regulates the activity of vinculin and talin and ultimately leads to integrin activation, adhesive patch formation, enhanced cytoskeletal junctions, and mechanical signaling (Calderwood, 2004).

Recent studies have shown that the presence of kindlin promotes integrin activation by talin. Kindlin has a PTB structure similar to that of talin and can bind simultaneously with talin in different motifs of integrin β (Figure 5B). Inhibition of kindlin binding to integrin inhibits integrin activation, and conversely, coexpression of kindlin and talin promotes integrin activation. Specifically, all kindlin isoforms bind to the membrane distal NxxY motif in the cytoplasmic tail of the integrin β subunit *via* the F3 substructural domain at the PTB site, leading to conformational changes and activation of the integrin receptor (Chen et al., 2019).

Piezo1 also plays an important role in mechanical signaling. Our study showed that mechanical stretching (CMS) increased Piezo1 expression and activation in human dermal fibroblasts (HDFs) (He et al., 2021). In erythropoiesis, activation of Piezo1 leads to Ca^2+^ inward flow. Ca^2+^-dependent protein kinase C (PKC) is activated and subsequently activates the small GTPase Rap1. Rap1 is activated through the interaction of the Rap1-interacting adapter molecule (RIAM) and talin, ultimately leading to integrin activation (Aglialoro et al., 2020) (Figure 5B).

The article "Extracellular matrix stiffness—The central cue for skin fibrosis" was published in 2023. Journal: Front Mol Biosci.

#### 4.2.1 FAK-mediated signal transduction

FAK, a tyrosine kinase with a binding domain with talin, can be recruited by paxillin to adhesion plaques and promote their homodimer formation (Mitra et al., 2005). The FAK Tyr397 site in the homodimer is autophosphorylated, which enhances binding to Src and a conformational change (Brami-Cherrier et al., 2014). In this FAK-Src complex, Src can transphosphorylate specific sites of FAK. Further phosphorylation of FAK exposes binding sites for Src homology 2 (SH2) domains and can further recruit Grb2 and PI3K (Mitra and Schlaepfer, 2006). Grb2 can further recruit SOS and activate the Ras/Raf/MEK/ERK signaling pathway (Figure 5B). PI3K binding to Src can activate the PI3K/AKT signaling pathway (Bolós et al., 2010) (Figure 5B). In addition, FAK regulates Rho GTPase activity, which leads to cytoskeletal remodeling and mediates directional cell movement (Tomar and Schlaepfer, 2009). FAK increases the expression of cellular myogenic markers and epithelial cell migration through the small G protein Cdc42 (Han et al., 2011; Wen et al., 2022). These signaling pathways are also present in TGF-β signaling (Figure 6). G proteins and small G proteins regulate FAK activity. Protein-activated receptor 1 (PAR1) and sphingosine-1-phosphate receptor 1 (S1P1) can upregulate FAK *via* downstream G protein activity (Thennes and Mehta, 2012).

FAK inhibitors reduce bleomycin-induced pulmonary fibrosis in mice (Zhao et al., 2016). Gurtner’s team showed that physical forces regulate fibrosis through the inflammatory FAK/ERK/MCP-1 pathway and that targeted inhibition of FAK inhibits mechanical force-induced hypertrophic scar formation (Wong et al., 2012).

#### 4.2.2 ILK-mediated signal transduction

Integrin-linked kinase (ILK) is another key node in integrin signaling (Legate et al., 2006). ILK, which is believed to be a pseudokinase, cannot phosphorylate any substrate directly (Boudeau et al., 2006; Byrne et al., 2017). ILK, PINCH, and parvin form a heterotrimeric complex, ILK-PINCH-PARVA (IPP). IPP is recruited to the adherent patch and acts as a hub for the integrin signaling network (Figure 5B). The complex connects the ECM to the actin cytoskeleton and protects ILK from proteasomal degradation (Legate et al., 2006). The ILK pathway is extensively involved in regulatory processes such as cell adhesion, apoptosis, proliferation, and migration (Martucci et al., 2021). In cancer, ILK promotes EMT and enhances the migration and invasion of cancer cells (McDonald and Dedhar, 2022). These cellular metabolism and behavior changes are facilitated by the activation of downstream signaling pathways such as AKT, Hippo, Wnt, and GSK-3β (Martucci et al., 2021). ILK can promote the transition from fibroblasts to myofibroblasts in the dermis with the transcription factor Snail1/Slug (Zoppi et al., 2018). The ILK-PI3K/AKT pathway regulates fibroblast migration (Li et al., 2016b).

The article "Extracellular matrix stiffness—The central cue for skin fibrosis" was published in 2023. Journal: Front Mol Biosci.

#### 4.2.3 Hippo signaling pathway

The Hippo pathway is an evolutionarily highly conserved signaling pathway that plays key roles in organ development, epithelial homeostasis, tissue regeneration, wound healing, and immune regulation (Dey et al., 2020). Many of these actions are mediated by the transcriptional effectors YAP and TAZ. The NDR (nuclear Dbf2-related) kinase family members LATS1 (large tumour suppressor 1) and LATS2 (large tumour suppressor 2) are major regulators of YAP/TAZ. Many upstream proteins are involved in the regulation of LATS activity. These include the integrins mentioned earlier and TGFβ-related signaling proteins such as ILK, FAK-Src, and Rho (Piersma et al., 2015; Dey et al., 2020) (Figure 5B). In addition, YAP/TAZ can directly transduce mechanical signals of the ECM independently of the Hippo/LATS cascade (Figure 5B). This process requires the involvement of Rho GTPase and the tension of the actin cytoskeleton (Dupont et al., 2011). Notably, increased ECM stiffness can reduce DNA methylation in the promoter region of YAP, suggesting an epigenetic role of mechanical signaling in cellular alterations (Jang et al., 2021). YAP/TAZ can regulate the expression of profibrotic genes through TEAD transcription factors, specifically CTGF, PAI-1, and LOX (Dey et al., 2020). A clear and complete description of the Hippo/YAP signaling network was previously reviewed by Rognoni and Walko (Rognoni and Walko, 2019).

## 5 Current therapeutic strategies and future perspectives

Skin fibrosis and scar formation are common outcomes of surgery, pathological injury and some diseases. They are characterized by myofibroblast proliferation and ECM deposition that result in mechanical stiffness modulation. Basic and clinical research has shown that a variety of treatments are available for patients with skin fibrosis and scar formation, including surgical, drug and combination treatments. Although some existing drugs have been preliminary proved the efficiency in skin fibrosis, there is still a long way to develop a satisfied therapy (Kothari et al., 2019). Targeted therapies can significantly reduce side effects and improve the efficacy of treatment. With the in-depth study of the molecular mechanisms of skin fibrosis, molecular targeted therapy will become the key direction of skin fibrosis. The inhibition of TGF-β and integrin pathways are important in targeted therapies. Upregulation of MMP expression or activity is also a valuable direction. In addition, new therapeutic approaches, such as RNA and stem cell transplantation, have emerged.

The article "Extracellular matrix stiffness—The central cue for skin fibrosis" was published in 2023. Journal: Front Mol Biosci.

### 5.1 Targeted inhibition of TGF-β signaling pathway

As previously mentioned, TGF-β, a profibrotic factor controlled by mechanical stress and inflammatory factors, plays an important role in the physiopathological events of skin fibrosis and has become a central target for pharmacological intervention (Batlle and Massagué, 2019). TGF-β1 overexpression in keratin-forming cells induces skin inflammation, and significant epidermal hyperplasia occurs. The TGF-β1/Smad3 signaling pathway is activated during skin photoaging and induces the production of MMPs, leading to increased collagen type I and ECM deposition (Fisher et al., 2016). Recessive dystrophic epidermolysis bullosa (RDEB) is an inherited skin disease characterized by increased mechanical fragility of the skin. A comprehensive gene expression study by Knaup showed that untransformed RDEB keratinocytes also display elevated levels of TGF-β1, which affects the expression levels of collagen type VII (Knaup et al., 2011). Patients with SSc have extensive skin fibrosis and visceral organ involvement, for which the TGF-β signaling pathway is often thought to be the main mechanism (Verrecchia et al., 2006; Sargent et al., 2010). In SSc patients, TGF-β promotes myofibroblast differentiation by stimulating the expansion of KLRG1-ILC2s (natural ILC2s) and reducing IL10 production. Thus, TGF-β signaling pathway is an important therapeutic target in skin fibrosis.

Targeted ablation of TGFBR2 in mice induces the overproliferation of keratin-forming cells induced by external factors (Guasch et al., 2007). Han’s study demonstrated that the degree of skin inflammation was associated with TGF-β1 expression, and Enbrel and Rosiglitazone, an effective treatment for human psoriasis, can effectively alleviate skin inflammation (Han et al., 2010). The application of pirfenidone and IL10 combination therapy significantly reduced skin fibrosis in the SSc mouse model (Laurent et al., 2021). Rituximab (RTX) may improve skin and lung fibrosis in SSc patients *via* the TGF-β-Dkk-1 axis (Daoussis et al., 2016). Additionally, overexpression of TGF-β at different sites may have different effects. Acute induction of TGF-β1 overexpression in the suprabasal layer of the epidermis reduced epidermal overproliferation in the skin, whereas sustained induction of TGF-β1 overexpression in the basal layer did not cause significant changes in the epidermis (Wang et al., 1999). TGF-β can stimulate cancer-associated fibroblasts (CAFs) to play an important role in regulating the tumor ECM (Chen and Song, 2019). In addition, the treatment of fibrosis in other tissues may also inform the treatment of skin fibrosis. The small-molecule inhibitor pirfenidone has been approved for the treatment of pulmonary fibrotic disease (Behr et al., 2021). In lung fibroblasts, pirfenidone can significantly inhibit TGF-β1-stimulated fibroblast-mediated collagen gel contraction, migration, and collagen triple helix repeat containing protein 1(CTHRC1) release. CTHRC1 is able to activate fibroblasts and recruit M2 macrophages (Jin et al., 2019). Buserelin and oleuropein have been shown to reduce fibrosis in the lung and kidney in mouse models (Akhurst and Hata, 2012). However, their use in cutaneous fibrosis is still being explored.

The article "Extracellular matrix stiffness—The central cue for skin fibrosis" was published in 2023. Journal: Front Mol Biosci.

Oxidative stress is influenced by TGF-β, which has shown a large role in the pathogenesis and treatment of dermal fibrosis. TGF-β activates several oxidative stress-related genes involved in the profibrotic pathway, acting through Smad and non-Smad pathways to enhance fibroblast recruitment and differentiation, leading to ECM deposition (Akhurst, 2012; Liu et al., 2012). A study of dermal fibroblasts from patients with scleroderma showed that following the application of antioxidants with oxidative stress inhibition, ERK1-2 and NF-kB activity reduced ECM deposition (Shroff et al., 2014). Similarly, simvastatin, arsenic trioxide and (PHTE) (Do and Eming, 2016)NQ have been shown in preliminary experiments to prevent skin fibrosis (Kavian et al., 2012; Bagnato et al., 2013). MMP exposure can also increase oxidative stress and stimulate fibroblast differentiation (Radisky et al., 2007). In summary, Oxidative stress is a potential target in skin fibrosis treatment.

Targeting the expression of genes downstream of the TGF-β1 signaling pathway, such as p53 and Smad3 and TGF-β1 oxidative stress-dependent genes, has also emerged as a therapeutic option for skin fibrosis (Samarakoon et al., 2013). Ebselenolide and enthesopine have been shown to reduce fibrosis in the lung and kidney in a mouse model (Shroff et al., 2014). In irradiated mice, exogenous interleukin 1β (IL1B) induces IL1B mRNA expression and rapidly increases MMPs but fails to reduce IL1-associated collagen accumulation (Liu et al., 2006).

### 5.2 Targeted degradation of ECM *via* MMP

MMP acts directly on the ECM and is regulated by mechanical stress and inflammatory factors involved in the proliferation of the ECM. Therapeutic studies targeting MMP have demonstrated its effectiveness to some extent. It has been shown that expression of MMP activity during wound healing can inhibit scar formation and may reduce fibrosis during healing. In most cases, MMP shows profibrotic activity, and MMP inhibitors may potentially treat fibrosis (Radisky et al., 2007). Core proteoglycans can treat pathological skin fibrosis by upregulating the expression of MMP-1 and MMP-3 mRNAs and decreasing the expression of collagen type I and type III mRNAs (Lee et al., 2015). After treatment with bone marrow mesenchymal stem cell (BM-MSC) transplantation, lesioned skin showed decreases in TGF-β1 and α-smooth muscle actin-positive cells, increased MMP expression, attenuated myofibroblast proliferation and ECM deposition, and collagen alignment similar to that of normal skin (Gourdie et al., 2006; Wu et al., 2014). MMP activation reduces excessive collagen deposition and subsequent scar formation to treat skin fibrotic disease (El Ayadi et al., 2020).

The article "Extracellular matrix stiffness—The central cue for skin fibrosis" was published in 2023. Journal: Front Mol Biosci.

However, excessive activation of MMPs can lead to excessive hydrolysis of collagen, which can lead to safety risks such as bleeding, organ perforation or rupture. This requires special attention in the antifibrotic treatment of organs such as the lungs, liver, kidneys and intestines. In contrast, the skin, the largest organ in the body, has high regenerative and compensatory capacities, providing a wider margin of safety for the use of MMPs to degrade the overproduced ECM in fibrosis areas. Even when extreme cases are considered, the excessive degradation of the ECM in areas of skin fibrosis could not pose a risk to the patient’s life.

### 5.3 New insights in skin fibrosis treatment by non-coding RNA

There is now a new understanding of the role of RNA in skin fibrosis. miRNAs are a group of small non-coding RNAs involved in skin fibrosis, including transforming growth factor-β signaling, ECM deposition, fibroblast proliferation and differentiation. There are both pro- and antifibrotic miRNAs. Antifibrotic miRNAs can be upregulated in treating skin fibrosis using mimetics and viral vectors. Conversely, profibrotic miRNAs can be downregulated using anti-miRNAs (Babalola et al., 2013). Since miR-486-3p mediates the overexpression of K17 protein under the regulation of the TGF-β/Smad pathway, thereby inducing glial cell proliferation, activating miR-486-3p may be a potential therapeutic approach for psoriasis (Jiang et al., 2017).

## 6 Conclusion

Although the molecular mechanisms of skin fibrosis have been extensively studied, the *in vivo* situation is complicated by the interplay of signaling networks, genetic-environmental interactions and variations in individual susceptibility. This makes it challenging to obtain similar results in clinical trials, and ultimately, only a small proportion can be successfully translated into therapeutic approaches. Interactions between different systemic signals have received increasing attention in the pathogenesis and progression of the disease. New research areas have been proposed to study mechano-immune and neuro-mechanical signaling networks. Exploring signaling cross-talk from the perspective of these areas may lead to discoveries in the pathogenesis of cutaneous fibrosis. To better mimic the *in vivo* microenvironment, three-dimensional cell cultures are now often used for *in vitro* studies of biomechanical mechanisms. However, the matrix materials currently available for cell culture may be cytotoxic and have limitations in terms of their mechanical properties. Material improvements for three-dimensional cell culture or the development of novel matrix materials may contribute to breakthroughs in biomechanical studies of fibrosis.

The article "Extracellular matrix stiffness—The central cue for skin fibrosis" was published in 2023. Journal: Front Mol Biosci.

ECM stiffness, a central cue in the skin fibrosis process, may be an important factor to focus on in targeted therapies for the treatment of skin fibrosis. Compared to other organs, multiple delivery methods such as local injection and gel application can be easier to use in skin tissue and have a wider safety margin. Studies have demonstrated that reducing ECM stiffness by inhibiting the cross-linking of ECM structural proteins or causing appropriate hydrolysis of ECM can improve skin scarring. Targeted inhibition of the signaling pathways of TGF-β is also a valuable treatment therapy. Recently, a broader view of biological events, such as epigenetic and post-transcriptional regulation, may contribute to a deeper understanding of the mechanisms of skin fibrosis.

## Author’s Note

Figures were created with the authorization of Biorender.com.

## Glossary

ADAM: a disintegrin and metalloproteinase
APC: antigen-presenting cell
BCR: B cell receptor
BioF: biomechanical force
BM: basement membrane
BMM: bone marrow-derived macrophage
BM-MSC: bone marrow mesenchymal stem cell
CAF: cancer-associated fibroblasts
CMS: mechanical stretch
Co-Smad: co-chaperone Smad
CTGF/CNN2: connective tissue growth factor
DC: dendritic cell
ECM: extracellular matrix
EMT: epithelial-mesenchymal transition
ERK: extracellular signal-regulated kinase
FACIT: fibril-associated collagens with interrupted triple helices
FAK: focal adhesion kinase
GAG: glycosaminoglycan
GAP: GTPase-activating protein
GEF: guanine nucleotide exchange factor
HDF: human dermal fibroblast
HFUS: high-frequency ultrasound
IFN: interferon
IL: interleukin
IL1B: interleukin 1β
ILK: integrin-linked kinase
IPP: ILK-PINCH-PARVA
I-Smad: inhibitory Smad
ITGB1: integrin β1
JNK: c-Jun-N-terminal kinase
LAP: latency-associated peptide
LOX: lysyl oxidase
MAPK: mitogen-activated protein kinase
MAPKK/MEK: mitogen-activated protein kinase kinase
MAPKKK: mitogen-activated protein kinase kinase
MMP: matrix metalloproteinase
MSC: mesenchymal stem cell
mTOR: mammalian target of rapamycin
mTORC: mTOR complex
NDR kinase: nuclear Dbf2-related kinase
NFAT: nuclear factor of activated T cells
LATS: large tumour suppressor kinase
NF-κB: Nuclear factor kappa-B
OCT: optical coherence tomography
OPN: osteopontin
PAR1: protein-activated receptor 1
PAK2: p21-activated kinase 2
PD: papillary dermis
PDGF: platelet-derived growth factor
PKC: protein kinase C
RD: reticular dermis
RDEB: recessive dystrophic epidermolysis bullosa
RGD: sequence Arg-Gly-Asp
RIAM: Rap1-interacting adapter molecule
ROCK: Rho-associated coiled-coil-containing protein kinase
R-Smad: receptor-regulated Smad
RTX: rituximab
RXFP1: relaxin family peptide receptor-1
S2P2: sphingosine-1-phosphate receptor 1
SH2: Src homology 2
SLRP: small leucine-rich proteoglycan
SSc: systemic sclerosis
TAK1: transforming growth factor-β-activated kinase 1
TAZ: transcriptional coactivator with PDZ-binding motif
TCR: T cell receptor
TGF-β: transforming growth factor-β
TGFBR: transforming growth factor-β receptor
TIMP: tissue inhibitors of metalloproteinase
TNF-α: tumor necrosis factor-α
YAP: yes-associated protein 1
